This article has been retracted.

# Effect Analysis of Epidural Anesthesia with 0.4% Ropivacaine in Transforaminal Endoscopic Surgery

**DOI:** 10.1155/2021/2929843

**Published:** 2021-10-06

**Authors:** Bingwei Hu, Hongwei Wang, Tingting Ma, Zhimei Fu, Zhiying Feng

**Affiliations:** ^1^Department of Pain, The First Affiliated Hospital, Zhejiang University School of Medicine, Hangzhou 310003, China; ^2^Department of Anesthesiology, Tongde Hospital of Zhejiang Province, Hangzhou 310012, China

## Abstract

**Background:**

Epidural anesthesia used in percutaneous endoscopic lumber discectomy (PELD) has the risk of complete neurotactile block. Patients cannot timely respond to the operator when the nerve is touched by mistake, so the potential risk of nerve injury cannot be avoided. According to pharmacodynamics, with the decrease of local anesthetic concentration, the nerve tactile gradually recovered; however, the analgesic effect also gradually weakened. Therefore, it is necessary to explore an appropriate concentration of local anesthetics that can keep the patients' nerve touch without pain. By comparing the advantages and disadvantages of 0.4% ropivacaine epidural anesthesia, local anesthesia and intravenous anesthesia on intraoperative circulation fluctuation, the incidence of salvage analgesia and the incidence of nerve non-touch, the feasibility of using low concentration epidural anesthesia in PELD to obtain enough analgesia and avoid the risk of nerve injury was confirmed.

**Methods:**

153 cases of intervertebral foramen surgery from October 2017 to January 2020 were selected and divided into local anesthesia group (LA group), 0.4% ropivacaine epidural anesthesia group (EA group), and intravenous anesthesia group (IVA group) according to different anesthesia methods. The changes of blood pressure and heart rate, the incidence of rescue analgesia and nerve root non-touch were compared among the three groups.

**Results:**

The difference of map peak value among the three groups was statistically significant (*P* < 0.001); pairwise comparison showed that the map peak value of the LA group was higher than that of the EA group (*P* < 0.001) and IVA group (*P* < 0.001), but there was no statistical significance between the EA group and IVA group. The difference of HR peak value among the three groups was statistically significant; pairwise comparison showed that the HR peak value of the LA group was higher than that of the EA group (*P* < 0.001) and IVA group (*P* < 0.001), but there was no statistical significance between the EA group and IVA group. There was significant difference in the incidence of intraoperative hypertension among the three groups (*P* < 0.05); pairwise comparison showed that the incidence of intraoperative hypertension in the EA group was lower than that in the LA group (*P* < 0.05), while there was no significant difference between the IVA group, EA group, and LA group. There was significant difference in the incidence of rescue analgesia among the three groups (*P* < 0.01); pairwise comparison showed that the incidence of rescue analgesia in the EA group was lower than that in the LA group (*P* < 0.05) and IVA group (*P* < 0.05), but there was no significant difference between the LA group and IVA group. Due to the different analgesic mechanisms of the three anesthesia methods, local anesthesia and intravenous anesthesia do not cause the loss of nerve tactile, while the incidence of nerve tactile in 0.4% ropivacaine epidural anesthesia is only 2.4%, which is still satisfactory.

**Conclusion:**

Epidural anesthesia with 0.4% ropivacaine is a better anesthesia method for PELD. It not only has a low incidence of non-tactile nerve, but also has perfect analgesia and more stable intraoperative circulation.

## 1. Introduction

Percutaneous endoscopic transforaminal lumbar discectomy (PELD) is easy to touch or injure the spinal cord and nerve due to its close proximity to the spinal cord and dural sac. In order to avoid nerve injury, PELD is mainly local anesthesia, or intravenous anesthesia, general anesthesia or epidural anesthesia by anesthesiologists [1, 2]. General anesthesia can provide perfect analgesia, but it is difficult to find nerve injury due to unconsciousness of patients [3–5]. Spinal nerve function monitoring [6, 7] can provide protection for avoiding nerve injury under general anesthesia. However, additional equipment, personnel, and medical costs limit the popularization of the technology. Although patients with local anesthesia retain consciousness, previous studies have shown that analgesia is insufficient [8], and various analgesic drugs are needed to remedy [9, 10]. Epidural anesthesia can also retain the consciousness of patients and provide perfect analgesia. The other advantage is that the motor function of the lower limbs of the patients remains when the concentration of local anesthetics is low. The surgeon can detect the nerve injury by observing the movement of the toes of the patients [5, 11]. However, this is not the indicator that the surgeon really wants. Because of the sensory motor separation characteristics of ropivacaine, although a certain concentration of ropivacaine retains the motor function, the sensory fibers are completely blocked (including pain and touch), and the patients cannot perceive that the nerve tissue is touched by mistake during the operation. Therefore, in theory, blocking pain and retaining touch is a reliable index to avoid nerve injury. Pain was mainly transmitted by myelinated a *δ* fibers (2–6 *μ*m) and unmyelinated C fibers (0.3–3 *μ*m), while touch was mainly transmitted by myelinated a *β* fibers (6–12 *μ*m). Different nerve fibers have different susceptibilities to local anesthetics. A *δ* nerve fiber is more susceptible to local anesthetics than a *β* nerve fiber, which leads to more pain block than touch [12]. Therefore, local anesthetics at appropriate concentrations can produce pain tactile separation block. Although some anesthesiologists [13] also recognize that low concentration of local anesthetics can retain the tactile sensation of nerve, there is no study to provide reference concentration of local anesthetics. Routine epidural anesthesia often uses 0.5% ropivacaine; although the analgesia is perfect, the nerve root tactile and lower limb motor function of patients are completely lost. Ren et al. [11] found that the analgesic effect of epidural anesthesia was satisfactory even when the concentration of ropivacaine was reduced to 0.375%. Therefore, when the concentration of ropivacaine is between 0.375% and 0.5%, there is an appropriate concentration, which can not only provide enough analgesia for patients but also retain nerve root tactile sensation. At this concentration, the patient's nerve root can be timely feedback when touched by mistake, and the operator can stop the operation in time to terminate the occurrence of nerve injury. Since October 2017, some patients with PELD in Zhejiang Litongde Hospital were treated with 0.4% ropivacaine epidural anesthesia, and the loss of nerve root tactile sensation was recorded in the electronic medical record.

## 2. Materials and Methods

### 2.1. Case Selection and Data Collection

Medical records of patients scheduled for PELD from October 2017 to January 2020 were collected from electronic medical record database (docare clinical anesthesia information system V5.0, madiston medical technology) of Zhejiang Litongde Hospital. Inclusion criteria were as follows: ASA grade I-II and patients scheduled for percutaneous transforaminal endoscopic discectomy. Exclusion criteria were as follows: age less than 18 or more than 80 years old; previous history of lumbar surgery; heart disease or cardiac insufficiency; liver and kidney dysfunction; patients with severe arrhythmia; patients with previous or current history of nervous system and mental disease; patients with abnormal coagulation function or platelet count; patients with other operations at the same time; and 2 or more segments of intervertebral disc nucleus pulposus removal. According to different anesthesia methods, they were divided into local anesthesia group (LA group), epidural anesthesia group (EA group), and intravenous anesthesia group (IVA group).

① Local anesthesia: 1% lidocaine infiltration anesthesia layer by layer. ② Epidural anesthesia with 0.4% ropivacaine: two segments of the lumbar spine were used as epidural puncture points on the cephalic side of the operation, and the epidural catheter was indwelled and placed toward the caudal side. After 5 minutes of 1% lidocaine test dose, 0.4% ropivacaine was given in batches until the anesthesia plane covered the operation area. ③ Intravenous anesthesia: 1 *μ*g/kg fentanyl was slowly injected after prone position, and dexmedetomidine loading dose was 1 *μ*g/kg (infusion time was 10 min), and then it was maintained at 0.3–0.5 *μ*g·kg^−1^·H^−1^ for no more than 30 min. ④ Remedial analgesia: simple use of opioid remedy can obtain enough analgesic effect, but there is a risk of respiratory depression; especially in prone position, it will greatly increase the difficulty of rescue. Therefore, according to the patient's pain performance, anesthesiologists implement individualized multimodal analgesia (non-steroidal, weak opioid, and strong opioid analgesics) to remedy the pain, so as to minimize the occurrence of drug side effects.

### 2.2. Evaluating Indicator

Eneral information of patients enrolled in the study in the database, including gender, age, hypertension, height, weight, body mass index, basic mean arterial pressure (basicmap) and basic heart rate (basichr) at admission. The historical records of intraoperative vital signs were displayed intensively (data collection interval was 1 min), the mean arterial pressure (premap, postmap) and heart rate (prehr, posthr) at the moment of entering the operating room and at the end of the operation, the peak intraoperative mean arterial pressure (intramap) and the peak intraoperative heart rate (intrahr), the incidence of additional analgesics due to intolerance of pain, and the time of operation were registered the amount of transfusion during operation. Intraoperative hypertension was defined as a 20% or more increase in peak mean arterial pressure (figure) compared with baseline map. The presence of nerve root sensation was recorded (whether there was radiating pain or swelling sensation in the innervated area when the operator touched the nerve root consciously).

### 2.3. Statistical Analysis

SPSS 25.0 was used for statistical analysis and Graphpad Prism 8 was used for mapping. For continuous data, the Shapiro–Wilk test was used to test the normality. The measurement data conforming to the normal distribution were described by means and standard deviation (mean ± SD), and one-way ANOVA was used; the measurement data not conforming to the normal distribution were described by median (M) and interquartile (Q), and Kruskal–Wallis *h* test of independent samples was used. The counting data were described as percentages, and the *χ*^2^ test was used. The Bonferroni method was used to correct the level of *α*. All tests were bilateral tests, and *P* < 0.05 indicated that the difference was statistically significant.

## 3. Result

In this study, 138 patients met the inclusion criteria, 15 patients met the exclusion criteria, and finally 123 patients were included in the study (Figure 1). There were 44 cases in the LA group, 41 cases in the EA group, and 38 cases in the IVA group. By the Shapiro–Wilk test, height, weight, BMI, basic map, basic HR, preoperative map, preoperative HR, intraoperative map peak, intraoperative HR peak, postoperative map, postoperative HR, and operation time were in normal distribution, and the data were analyzed by means of mean and standard deviation (mean* ± *SD). According to Levene's test of homogeneity of variance, the data were consistent with the homogeneity of variance; the age and infusion volume of patients in each group did not completely conform to the normal distribution, and the data were described by median (M) and interquartile (Q).

### 3.1. General Information

The height, weight, BMI, basic map, basic HR, and operation time of the patients were analyzed by one-way ANOVA. The Kruskal–Wallis *h* test of independent samples was used for age and infusion volume, and *χ*^2^ test was used for gender and history of hypertension. The results showed that there was no significant difference among the groups (Table 1).

### 3.2. Comparison of Mean Arterial Pressure of Three Anesthesia Methods during Perioperative Period

One-way ANOVA showed that there was no significant difference in map before and after operation, but there was significant difference in map peak value during operation (Welch ANOVA was used for uneven variance; Welch *F* = 9.828, *P* < 0.001). The Games–Howell test showed that the peak value of intraoperative map in the LA group was 18.4 mmHg higher than that in the EA group (95% CI: 8.5–28.3 mmHg), and the difference was statistically significant (*P* < 0.001); the peak value of intraoperative map in the LA group was 13.3 mmHg higher than that in the IVA group (95% CI: 2.3–24.0 mmHg), and the difference was statistically significant (*P* < 0.05); there was no statistical significance between the EA group and IVA group (Figure 2).

### 3.3. Comparison of Perioperative Heart Rate among Three Anesthesia Methods

There was no significant difference in HR before and after operation in each group by one-way ANOVA, but there was significant difference in HR peak during operation between groups (uneven variance, Welch ANOVA; Welch *f* = 24.166, *P* < 0.001). The Games–Howell test showed that the peak value of intraoperative HR in the LA group was 17.7 bpm higher than that in the EA group (95% CI: 11.6–23.7 bpm), and the difference was statistically significant (*P* < 0.001); the peak value of intraoperative HR in the LA group was 14.30 bpm higher than that in the IVA group (95% CI: 5.9–22.2 bpm), and the difference was statistically significant (*P* < 0.001); there was no statistical significance between the EA group and IVA group (Figure 3).

### 3.4. Comparison of the Incidence of Intraoperative Hypertension among Three Anesthesia Methods

The incidence of intraoperative hypertension in the LA group, EA group, and IVA group was 36.4%, 9.8%, and 18.4%, respectively. *χ*^2^ test showed that there was significant difference in the incidence of intraoperative hypertension among the three groups (*χ*^2^ = 9.175, *P* < 0.05). Pairwise comparison showed that there was significant difference between the LA group and EA group (*P* < 0.05), but there was no significant difference between the LA group and IVA group and EA group and IVA group (Table 2).

### 3.5. Comparison of the Incidence of Intraoperative Salvage Analgesia among Three Anesthesia Methods

The incidence of intraoperative salvage analgesia in the LA group, EA group, and IVA group was 43.2%, 12.2%, and 36.8%, respectively. *χ*^2^ test showed that there was significant difference in the incidence of intraoperative salvage analgesia among the three groups (*χ*^2^ = 10.456, *P* < 0.01) (Table 3). Pairwise comparison showed that there were significant differences between the EA group and LA group (*P* < 0.05) and EA group and IVA group (*P* < 0.05), but there was no significant difference between the LA group and IVA group (Table 3).

### 3.6. The Incidence of Non-Tactile Nerve Root in Three Anesthesia Methods

Because local anesthetics of LA mainly act on nerve endings to block the transmission of pain, while opioids of IVA mainly act on central opioid receptors to produce analgesic effect, neither of them can significantly affect the tactile sensation of nerve roots. EA not only blocked the pain fibers but also blocked the tactile fibers and motor nerves because of the action of local anesthetics on nerve roots and spinal cord. The degree of EA was positively correlated with the concentration of local anesthetics. In 41 patients undergoing epidural anesthesia with 0.4% ropivacaine, only one patient (2.4%) lost nerve root tactile sensation.

## 4. Discussion

To avoid nerve injury, local anesthesia with a low incidence of nerve root injury is usually recommended for PELD [14]. When a nerve is mistakenly touched, the patient can provide timely feedback. A study [3] showed that most patients with local anesthesia had moderate or severe pain when their nerve roots were stimulated, and 15 of 30 patients had fear of surgery. Therefore, anesthesiologists need to explore anesthesia methods that can not only provide effective analgesia, but also make the patient's feedback nerve be touched by mistake. Low-concentration ropivacaine epidural anesthesia is the most common research at present. It not only has good analgesic effect but also can preserve the motor function of patients' lower limbs. The operator can detect the nerve injury by observing the movement of patients' toes during the operation [5, 11]. But this method has a lag, and once the motor function is damaged, nerve damage occurs. Therefore, we need to find the local anesthetic concentration that can make the patient feedback the nerve touched immediately. 0.4% ropivacaine epidural anesthesia is a better choice, and only one of 41 patients in this study had complete loss of nerve root tactile. Because of the different mechanisms of action of drugs, 0.4% ropivacaine epidural anesthesia cannot completely retain the patient's nerve tactile, and only 2.4% of the incidence of nerve non-tactile is still satisfactory. The analgesic effect of epidural anesthesia is better than that of local anesthesia [15–18]. The analgesic effect of epidural anesthesia with 0.25% ropivacaine is close to that of local anesthesia [18]. In this study, the incidence of rescue analgesia in 0.4% ropivacaine epidural anesthesia was significantly lower than that in local anesthesia, which indicated that the analgesic effect of 0.4% ropivacaine epidural anesthesia was better than that of local anesthesia, which was consistent with previous studies. Moreover, pain often leads to cardiovascular events. However, the peak value of mean arterial pressure, peak value of intraoperative heart rate, and incidence of intraoperative hypertension in 0.4% ropivacaine epidural anesthesia were significantly lower than those in local anesthesia, and the probability of cardiovascular events was lower. Therefore, epidural anesthesia has advantages over local anesthesia in reducing intraoperative salvage analgesia and stabilizing circulation. Compared with intravenous anesthesia, the incidence of rescue analgesia in 0.4% ropivacaine epidural anesthesia is much lower. However, this does not mean that its analgesic effect is better than intravenous anesthesia. Because the analgesic effect of intravenous anesthesia depends on the dose of opioids, the analgesic effect of intravenous anesthesia in this study can be improved by increasing the dose of opioids, but in the case of patients with PELD in prone position, adverse reactions such as respiratory depression caused by excessive dose are often more difficult to deal with. Therefore, the analgesic effect of 0.4% ropivacaine epidural anesthesia is better when the dosage of intravenous anesthesia is lower, and the safety of 0.4% ropivacaine epidural anesthesia is higher when the dosage of intravenous anesthesia is higher.

In summary, PELD with 0.4% ropivacaine epidural anesthesia can retain the nerve touch to a large extent to avoid nerve injury. At the same time, its analgesic efficacy and safety are better than local anesthesia and intravenous anesthesia. However, the choice of local anesthetic concentration in the study is based on the clinical experience of anesthesiologists, and it is not clear whether epidural anesthesia can reach the lower limit of effective analgesia concentration and the upper limit of nerve root tactile retention concentration. According to pharmacodynamics, for patients, the local anesthetic concentration just reached the pain disappeared, that is, the minimum effective concentration (MEC); with the increase of local anesthetic concentration, there is a suitable concentration, the patient's nerve tactile just disappeared, that is, the maximum tolerable concentration (MTC) of the patient's nerve tissue tactile is retained (Figure 4). The concentration of anesthetics is in the effective range between MEC and MTC. When the operation touches the nerve, the innervated area often shows slight radiation pain or acid swelling. When the operator receives feedback from the patient, the operation is terminated in time to avoid nerve injury. Therefore, the following study will apply biased coin design (BCD) to explore MEC and MTC of ropivacaine in PELD.

## Figures and Tables

**Figure 1:** Patient flow diagram.

**Figure 2:** ^*∗*^The peak value of map in the LA group was significantly higher than that in the EA group (*P* < 0.001). ^*∗∗*^The peak value of map in the LA group was significantly higher than that in the IVA group (*P* < 0.05).

**Figure 3:** #The peak value of intraoperative HR in LA group was significantly different from that in EA group (*P* < 0.001); ##the peak value of intraoperative HR in LA group was significantly different from that in IVA group.

**Figure 4:** Dose effect curve of local anesthetics on pain, touch, and motor function.

**Table 1:** Information of patients.

Index	Group			Statistics	*P* value
	LA group	EA group	IVA group		
Sample size	44	41	38	—	—
Gender (example, %)					
Male	21 (7.7)	27 (53.7)	20 (52.6)	*χ* ^2^ = 2.977	0.226
Age (years, *M* (*Q*))	52.5 (26)	58 (24)	54.5 (13)	*H* = *2.199*	0.333
Height (cm, $\bar{x}\pm s$)	164.1 ± 7.6	166.8 ± 8.5	164.4 ± 7.0	*F* = *1.533*	0.220
Body weight (kg, $\bar{x}\pm s$)	63.3 ± 10.6	65.1 ± 12.9	63.0 ± 9.8	*F* = *0.432*	0.650
BMI (kg/m^2^, $\bar{x}\pm s$)	23.4 ± 2.4	23.2 ± 3.2	23.2 ± 2.6	*F* = *0.020*	0.980
Previous hypertension (cases, %)					
Yes	9 (20.5)	10 (24.4)	9 (23.7)	*χ* ^2^ = 0.479	0.787
BasicHR (times/min, $\bar{x}\pm s$)	73.2 ± 11.2	74.4 ± 9.1	75.4 ± 11.3	*F* = *0.458*	0.634
BasicMAP (mmHg, $\bar{x}\pm s$)	93.5 ± 11.3	93.1 ± 11.6	97.0 ± 13.6	*F* = *1.262*	0.287
Infusion volume (ml, *M* (*Q*))	725 (200)	700 (200)	700 (250)	*H* = *0.336*	0.845
Operation time (min, $\bar{x}\pm s$)	93.4 ± 19.9	93.1 ± 17.0	94.0 ± 23.4	*F* = *0.023*	0.980

**Table 2:** Comparison of the incidence of intraoperative hypertension among three groups.

Intraoperative hypertension	Grouping			Total	Statistic	*P* value
	LA group	EA group	IVA group			
Yes	16^a^	4^b^	7^a,b^	27	*χ* ^2^ = 9.175	0.010
Nothing	28	37	31	96		
Total	44	41	38	123		

There was significant difference in the incidence of hypertension among the three groups (*P* < 0.05); the Bonferroni method was used to correct the level of blood pressure between two groups, and there was significant difference between the EA group and LA group (*P* < 0.05).

**Table 3:** Comparison of the incidence of analgesic rescue.

Remedial analgesia	Grouping			Total	Statistic	*P* value
	LA group	EA group	IVA group			
Yes	19^a^	5^b^	14^a^	33	*χ* ^2^ = 10.456	0.005
Nothing	25	36	29	90		
Total	44	41	38	123		

There was significant difference in the incidence of intraoperative rescue among the three groups (*P* < 0.01); the Bonferroni method was used to correct the level of *α*, the difference was statistically significant between the EA group and LA group (*P* < 0.05), and the difference was statistically significant between the EA group and IVA group (*P* < 0.05).

## Data Availability

The simulation experiment data used to support the findings of this study are available from the corresponding author upon request.

## References

[1] Liu Y. M., Zhao S. M. (2018). Clinical research progress of percutaneous spinal endoscopy in the treatment of lumbar disc herniation. *Chinese Journal of Preventive Medicine*.

[2] Sairyo K., Chikawa T., Nagamachi A. (2018). State-of-the-art transforaminal percutaneous endoscopic lumbar surgery under local anesthesia: discectomy, foraminoplasty, and ventral facetectomy. *Journal of Orthopaedic Science*.

[3] Ye X.-F., Wang S., Wu A.-M. (2020). Comparison of the effects of general and local anesthesia in lumbar interlaminar endoscopic surgery. *Annals of Palliative Medicine*.

[4] Wu K., Zhao Y., Feng Z., Hu X., Chen Z., Wang Y. (2020). Stepwise local anesthesia for percutaneous endoscopic interlaminar discectomy: technique strategy and clinical outcomes. *World Neurosurgery*.

[5] Zhu Y., Zhao Y., Fan G. (2018). Comparison of 3 anesthetic methods for percutaneous transforaminal endoscopic discectomy: a prospective study. *Pain Physician*.

[6] Xia X., Zheng C., Nie C. (2017). Application value of soleus H reflex monitoring in percutaneous interlaminar endoscopic surgery under general anesthesia. *Chinese Journal of Spine and Spinal Cord*.

[7] Hu K., Xiong M., Wang Y., Jin X., Zhou Y. (2015). Application of neurophysiological monitoring in percutaneous endoscopic lumbar discectomy. *Chinese Journal of Spine and Spinal Cord*.

[8] Gibson J. N. A., Cowie J. G., Iprenburg M. (2012). Transforaminal endoscopic spinal surgery: the future ‘gold standard’ for discectomy? - a review. *The Surgeon*.

[9] Fan Y., Gu G., Fan G. (2017). The effect of preoperative administration of morphine in alleviating intraoperative pain of percutaneous transforaminal endoscopic discectomy under local anesthesia. *Medicine*.

[10] Wang Y., Liu X., Li Y., Che F., Ai D. (2019). Effect of preemptive analgesia with oxycodone on spinal endoscopic nucleus pulposus removal. *Chinese Journal of Preventive Medicine*.

[11] Ren Z., He S., Li J. (2020). Comparison of the safety and effectiveness of percutaneous endoscopic lumbar discectomy for treating lumbar disc herniation under epidural anesthesia and general anesthesia. *Neurospine*.

[12] Zhuang X., Zeng Y., Chen B. (2010). *Modern Anesthesiology*.

[13] Huang Y., Lin J., Tao G., Wei H., Hang Y. (2017). Efficacy analysis of lumbar disc herniation treated by transforaminal endoscopy under epidural anesthesia. *Chinese Journal of Preventive Medicine*.

[14] Teli M., Lovi A., Brayda-Bruno M. (2010). Higher risk of dural tears and recurrent herniation with lumbar micro-endoscopic discectomy. *European Spine Journal*.

[15] Chen H. T., Tsai C. H., Chao S. C. (2011). Endoscopic discectomy of L5-S1 disc herniation via an interlaminar approach: prospective controlled study under local and general anesthesia. *Surgical Neurology International*.

[16] Xu T., Tian R., Qiao P., Han Z., Shen Q., Jia Y. (2019). Application of continuous epidural anesthesia in transforaminal lumbar endoscopic surgery: a prospective randomized controlled trial. *Journal of International Medical Research*.

[17] Fang G., Ding Z., Song Z. (2016). Comparison of the effects of epidural anesthesia and local anesthesia in lumbar transforaminal endoscopic surgery. *Pain Physician*.

[18] Zhu Y., Zhao Y., Fan G. (2017). Comparison of the effects of local anesthesia and epidural anesthesia for percutaneous transforaminal endoscopic discectomy in elderly patients over 65 years old. *International Journal of Surgery*.

